The article "Sleep effects on breathing and respiratory diseases" was published in 2009. Journal: Lung India.

# Sleep effects on breathing and respiratory diseases

**DOI:** 10.4103/0970-2113.56345

**Published:** 2009

**Authors:** Sumer S. Choudhary, Sanjiw R. Choudhary

**Affiliations:** *Department of Pulmonary Medicine, Sleep Medicine, Critical Care, Shree Ramjevan Choudhary Memorial Hospital and Research Centre, Nagpur - 02, India*

**Keywords:** Asthma, COPD, neuromuscular, sleep

## Abstract

To understand normal sleep pattern and physiological changes during sleep, sleep and breathing interaction, nomenclature and scales used in sleep study, discuss the effect of rapid eye movements and non-rapid eye movements while sleep and to review the effects of obstructive and restrictive lung disease on gas exchange during sleep and sleep architecture.

## INTRODUCTION

Sleep is a basic biological function in human beings and is as important as having a natural balanced and proper diet for good quality of life. It still requires much awareness about the effects and adversities in different clinical conditions in both patients and treating physicians. Sleep disorder alters the nature of sleep, which in turn alters the breathing pattern, ventilation and gas exchange. This may result in amplification of the underlying disorders, and hence increase burden of the disease.

Some of the diseases are familiar to the clinician, such as sleep apnea, resulting in arousal from sleep that improves airway patency but results in daytime sleepiness. Some of the respiratory diseases may cause breathing failure without any obvious obstruction. It is important to realize that recovery from upper airway events in obstructive sleep apnea does not always require arousal.

## NORMAL SLEEP

Sleep is not only a decrease in the level of consciousness but a much more complex phenomenon. The initial work done by Rechtehaffen and Kales in 1968, on sleep and its effects on different diseases, has progressed to a great extent but still requires much to be done. The most important landmark in sleep science is the discovery of REM sleep and the realization that sleep occurs in stages of rapid eye movements (REM) and non-REM sleep. The basic rules for sleep staging were given in 1968 in Rechtschaffen and Kales manual for sleep stages.

Normal sleep is divided into two stages: Rapid eye movements (REM) and non-rapid eye movements (NREM), which is further divided into four stages.

These stages are distinguished on the basis of electroence phalogram (EEG), electromyogram (EMG) and electro-oculogram (EOG).

### Wake stage

In human beings, in the awake and relaxed states with eye closed, EEG shows predominantly alpha activity, especially over the occipital area. The EEG rhythm shows moderately low voltage, mixed frequency pattern. REM and eye blinks are seen on the EOG with the eyes open, while the chin EMG shows tonic activity.

The article "Sleep effects on breathing and respiratory diseases" was published in 2009. Journal: Lung India.

### Rapid eye movements sleep

This period of sleep is characterized by very rapid eye movement, and resembles wakeful pattern but has greatly reduced muscle activity. It generally represents dreaming activity. This part of sleep is associated with the greatest respiratory and cardiac instability. The EEG in REM sleep is often referred to as desynchronized or activated. The activity is essentially low-voltage mixed-frequency pattern. There are two essential features that differentiate REM sleep from stage 1. The EEG shows saw tooth waves, and notched appearance that is best seen over the vertex.

### Non-rapid eye movements sleep

Classified into four stages according to the changes seen in EEG.

#### Stage 1

Relaxed wakefulness state with closed eye, exhibit alpha activity in EEG. Disappearance of this alpha activity is seen in this stage and the patient can be easily aroused. Vertex sharp waves are typical of stage 1 sleep, which are for short duration.

#### Stage 2

Appearance of K complexes (large biphasic waves) and sleep spindles is seen in this stage. These two features are characteristic of stage 2. K complexes should last at least 0.5 second and may have sleep spindles superimposed on the wave form.

#### Stages 3 and 4

Appearance of delta waves (large amplitude waves). This stage constitutes the deepest sleep. The percentage of delta wave declines with increasing age. In stage 3, slow waves with a frequency of <2 Hz are present for 20% to 50% of the epoch. In stage 4, such an activity is present in >50% of the epoch.

Delta Waves: <4Hz, 150-250 V

Theta Waves: 4-8 Hz, 100-200 V

Alpha Waves: 8-13 Hz, 50-100 V

Beta Waves: >13Hz, <50 V

As the sleep progresses from stage 1 to 4, the voltage increases and the frequency decreases. Waves on the EEG record are analyzed based on their frequency in Hertz or waves per second and voltage amplitude in microvolt or wave size, measured from trough to peak.

Normal individuals fall asleep within 20 minutes after going to bed and entering the successive stages of sleep, with REM occurring at about 90-100 minutes. Initially, deeper NREM occurs in the first half of sleep with more REM in the second half of sleep.

## ASSESSMENT OF SLEEP

Sleep assessment is conducted by overnight polysomno graphy usually with 8-hour duration recording. Multiple Sleep Latency Test (MSLT) can be conducted for assessing daytime sleepiness.

Conventional method of recording at sleep center

In this method, the patient has to sleep in the laboratory where the test is to be performed. The patent is made comfortable and a complete sleep test is performed using all the recommended channels.

The article "Sleep effects on breathing and respiratory diseases" was published in 2009. Journal: Lung India.

Multiple sleep latency test and maintenance of wakefulness test

This test is performed in patients with daytime sleepiness. The patient stays for a series of 4-5 daytime nap. MSLT and MWT are recorded in the same way, except, in MSLT the patient stays in the bed and is asked to sleep, whereas in MWT the patient is semi-reclining and asked to try to stay awake.

Portable home recording

There are a number of companies promoting their equipment for portable home recording without validation of the equipment. Simply performing the test without adequate examination and knowledge by the technician at home mostly gives fallacious reports. “The use of portable monitoring devices is not recommended for general population screening or in the absence of a pretest probability of the patient having a diagnosis of OSA, for the complaints other than OSA, without review of data interpretation, by physicians without familiarity with their use and limitations, and without trained personnel to perform technical scoring.”

The interpretation of sleep study begins with staging the record, in which the recorded sleep is reviewed and stages of sleep determined throughout. The single most important recording for sleep staging is the EEG.

## PHYSIOLOGICAL CHANGES DURING SLEEP

The true function of sleep till date remains a mystery; however, its physiological consequences that affect the body system are known. It affects temperature regulation, autonomic nervous system, cardiovascular system, respiratory system, immune system, gastrointestinal, renal system and reproductive system.

### Autonomic nervous system

Onset of sleep and NREM is characterized with increased parasympathetic and decrease sympathetic tone. In REM sleep, during Tonic REM (no eye movements) further increase in above features is observed. In Phasic REM (eye movements) increase sympathetic activity is observed, which occurs in bursts.

### Body temperature

During sleep there is decrease in the thermal setpoint, and the body temperature decreases by 1°C-2°C. Thermoregulation is maintained during NREM sleep but its response tends to be attenuated during REM sleep.

### Hormonal

Most hormones follow circadian and ultra-radian rhythm. Adrenocorticotropic hormone and cortisol secretion peaks between 4 and 8 am. Thyroid-stimulating hormone secretion is low during the day, increases in evening and peaks in the night before sleep.

### Cardiovascular

Cardiovascular system is dominated by parasympathetic activity. Increase in the vagal activity leads to electrical stability and decreased risk of arrhythmia. Accordingly, heart rate, blood pressure, stroke volume, cardiac output and systemic vascular resistance decrease. There is transient increase of 35% in heart rate in phasic REM sleep. Increased autonomic nervous system activity during REM sleep may increase the risk ventricular arrhythmia or exacerbate underlying pathology.

The article "Sleep effects on breathing and respiratory diseases" was published in 2009. Journal: Lung India.

### Respiratory

Transitions from wake state to NREM sleep, withdrawal of wakefulness drive results decrease in minute ventilation. There is progressive reduction in central respiratory drive through stage 1 to 4 of NREM Sleep. PaCO_2_ increases by 3-7 mmHg. During NREM the respiration is regular and predominantly under metabolic control as opposed to REM sleep, when respiration becomes irregular and depends on behavioral factor. Hypoxia and hypercapnic ventilatory responses fall on transition from wakefulness to NREM sleep and further depresses during REM sleep.

## NOMENCLATURE AND SCALES USED IN SLEEP STUDY

### Apnea

Cessation of airflow lasting 10 seconds or more.

### Hypopnea

Decrease in airflow latency 10 seconds or more generally defined as 50% decrease in flow accompanied by arousal or oxygen desaturation.

### Apnea index

Average number of apnea occurring during 1 hour of sleep.

### Apnea hypopnea index

Average number of apnea and hypopnea during 1 hour of sleep.

### Questionnaire to evaluate daytime sleepiness

In patients with complaint of excessive daytime sleepiness, the Stanford and Epworth Sleepiness Scale [Table 1] may be used to assess the severity of the symptoms of excessive sleepiness.

**Table 1:** Epworth sleepiness scale

Sitting and reading	0-3
Watching television	0-3
Sitting inactive in a public place (eg, a theatre or meeting)	0-3
As a passenger in a car for an hour without a break	0-3
Lying down to rest in afternoon	0-3
Sitting and talking to someone	0-3
Sitting quietly after lunch (when you have no alcohol)	0-3
In a car, while stopped in traffic	0-3

0 = would never doze, 1 = slight chance of dozing, 2 = moderate chance of dozing, 3 = high chance of dozing, Total score > 10 is considered abnormal

### Terminology for common sleep-related breathing disorders

Primary Central Apnea in adults or infants is a condition in which central sleep apnea occurs inherently due to electrical instability in the brain. Central sleep apnea as described in the Table 2 is due to certain precipitating conditions, few of which are highlighted in the Table given above. Alveolar hypoventilation may be idiopathic resulting in sleep related non-obstructive apnea or congenital central. The American Sleep Disorder Association Classifies OSA as given below:

**Table 2:** Current terminology for common sleep-related breathing disorders

Primary central apnea
Central sleep apnea: Cheyenne stroke breathing, high altitude periodic
breathing, drugs (barbiturates, morphine, etc), medical conditions
(hypothyroidism, renal failure, etc)
Primary sleep apnea of infancy
Obstructive sleep apnea
Sleep-related non-obstructive alveolar hypoventilation; idiopathic
Congenital central alveolar hypoventilation syndrome

Mild - OSA AHI 5-15

Moderate - OSA AHI 15-30

Severe - OSA AHI >30

The article "Sleep effects on breathing and respiratory diseases" was published in 2009. Journal: Lung India.

## EFFECTS OF SLEEP ON RESPIRATION

Sleep in normal course to a certain extent impairs breathing in normal individual. Gas exchange is impaired with a 2- to 8-mmHg increase in CO_2_ level. Pharyngeal muscle relaxation during sleep increases the upper airway resistance. Upper airway reflex dilator response is impaired during sleep and ventilator response to mechanical load may be blunted or absent. Recumbency and sleep decreases oxygen stores in the body and sleep depresses response to hypoxia and hypercapnia. Sleep induces hypotonia in upper airways, resulting in decrease and delayed response to negative pressure. Mortimore and Douglas have compared the response of upper airways pressure in normal and SAHS patients, and found that the latter have improved response to negative airway pressure.

Sleep exaggerates instability in breathing pattern. Periodic breathing is promoted by hypocapnia resulting from sustained hyperventilation at high altitude or pulmonary venous congestion that accompanies heart failure. The periodic breathing pattern are related to the characteristics of the lung chemoreceptor feedback loop and promoted by loss of behavioral override and low lung volumes. The periodic breathing mechanism is amplified by delay circulation time in heart failure and high ventilatory drive, caused by both hypoxia of high altitude and pulmonary congestion in heart failure.

Regular breathing periodicity in heart failure is restricted to stages 1 and 2 of NREM. Once periodic breathing in obstructive sleep apnea is initiated, mixed apnea may occur with both central and obstructive component. Hence, periodic breathing promotes obstructive sleep apnea. Similarly, ventilatory overshoots in obstructive sleep apneas cause central apneas.

REM has specific effects on breathing, with variability in breathing pattern and rib cage inhibition most often marked during phasic REM. The variability in breathing during REM is random and may be linked to cortical rather than chemoreceptor effects.

In normal subjects, in REM sleep normally decreases the tidal volume and ventilation and the effects are exaggerated to a great extent in patients with obstructive sleep apnea and respiratory disease. There is a large biological variability in the effect of REM sleeps on breathing and rib cage inhibition. Experimental hypercapnia results in more substantial inhibition of ventilation during REM and provides an additional possible mechanism for profound effects of REM in respiratory failure.

The article "Sleep effects on breathing and respiratory diseases" was published in 2009. Journal: Lung India.

Diurnal variation in symptoms of asthmas suggests that sleep and circadian rhythms influence pathophysiological mechanism in asthma.

Morning decrease in peak flow correlates with several mediators in asthma, inclusive of epinephrine, cortisol and histamine. In patients with nocturnal asthma, inflammatory response shows diurnal variation in eosinophilia. Recently, hypothalamic pituitary adrenal axis dysfunction and elevated melatonin have been implicated in nocturnal asthma.

In addition, to circadian influence specific sleep stage may also contribute. One series showed highest airway resistance in the lung in asthma that occurred during slow wave sleep.

## EFFECTS OF RESPIRATORY DISORDERS ON SLEEP

Many medical conditions are associated with insomnia or perception of disruption in the continuity of sleep. Elevated interleukin-4 and interleukin-B in patients with allergic rhinitis correlate with increased latency of REM and decreased REM. Patients with lung disease, chest wall restriction and neuromuscular diseases often have abnormalities in sleep and breathing during sleep. They have poor sleep quality, frequent arousals, hypoxia and hypercapnia.

### Obstructive pulmonary disease

It includes reversible airway disorders as seen in asthma, chronic obstructive lung disease, and chronic upper airway obstruction due to vocal cord paralysis. Upper airway obstruction associated with inspiratory stridor may mimic obstructive sleep apnea, with the exception that it does not reverse during day time. Prolonged desaturation occurs typically in REM and is associated with decrease tidal volume. In severely hyperinflated patients with COPD, having flat diaphragm, the occurrence of severe gas exchange abnormality is predicted by time spent in REM. In COPD, hypoxemia is more during sleep as compared to wakeful pattern. During sleep, increased hypoxemia is seen in REM sleep. The major cause is hypoventilation, increased ventilation perfusion mismatching and decrease in FRC.

A majority of patients with COPD have worsening respiratory failure, rather than obstructive sleep apnea. It was noted in two case series of severe COPD that 80% patients had sleep-associated desaturation. Hypoventilation with hypercapnia has been most consistently associated with the presence of desaturation in patients with COPD. In a series, of 54 patients with severe COPD, hypercapnia defined as >10 mmHg increase in sleep pCO_2_, for more than 20% of sleep was present in 43% of patients. Accumulation of secretion, patients of COPD, showed increased frequency of arousal and decreased total sleep time. In one of the cross-sectional study of symptomatic patient with COPD, 53% of patients reported insomnia and 23% complained of daytime sleepiness.

The article "Sleep effects on breathing and respiratory diseases" was published in 2009. Journal: Lung India.

Asthma patients have worsening of symptoms during night. Emergency room visits are more common at night. A study reports that maximum deaths due to asthma occur between 6 pm and 3 am. Airway function declines during night, whether the patient sleeps or not, though the decline is exaggerated by sleep. Hence, sleep may be one of the important factors in night-time desaturation and asthma exacerbation.

### Restrictive Lung Disorders

Heterogeneous group that limits lung expansion are termed as restrictive lung disorders. Common diseases include pleural diseases, neuromuscular disorders, scoliosis, parenchymal lung disease and massive obesity. Parenchymal lung disease increases ventilatory drive and dyspnea by neural mechanism, whereas other forms increase work of breathing. Similar to obstructive lung disease, a restrictive lung disorder interrupts the continuity of sleep and produce sleep-related hypoventilation and or hypoxemia. Schonhofer and Kohler showed that chronic ventilation for 12 months resulted in improvement in oxygen saturation during REM (25%) and NREM (+21), a 54% decrease in awakening and 18% improvement in sleep efficiency in a heterogeneous group of 15 patients with restrictive disorders. Ventilatory support in restrictive disorders improves daytime sleepiness, daytime hypoventilation, chronic respiratory muscle weakness, exercise endurance and pulmonary hemodynamics.

### Hypoventilation Syndromes

Patients with obstructive or restrictive pulmonary disease may experience hypoventilation that reflects mechanical restraint on ventilation as well as effects on dead space increase CO_2_ production in pulmonary diseases. Such patients experience excessive efforts in breathing as dyspnea in wake state and increased hypercapnia during sleep. Patients whose response to hypercapnia is blunted or those whose set point for paCO_2_ is increased, experience less dyspnea during wake situations and yet have increased hypercapnia during day time and increase more during night time. Some degree of ventilator reserve may be inferred by the ability to voluntarily lower paCO_2_ during day and by daytime improvement in hypoventilation when ventilation is supported during the night.

## CONCLUSION

There is substantial interaction between sleep and respiratory diseases, resulting in permissive effects of sleep on respiratory failure, bronchoreactivity, and mucous retention. Similarly, there is a negative effect of respiratory diseases on sleep quality and continuity. Hence, in any sleep study, measures of only apnea-hypoapnea index are most often inappropriate. Any sleep study should always be accompanied by measurement of components such as oxygen saturation, EOG, ECG, EMG and body position, with recording EEG. The EEG recording would certainly to an extent would help to identify the sleep quality and effects of various disease conditions in sleep cycles. In REM phase of sleep, rib-cage inhibition is observed. The respiratory variability is due to cortical effect. Chronic ventilation improves the patient's oxygen saturation in both REM and NREM phases of sleep, less frequency of awakening in night and improves sleep efficiency.

The article "Sleep effects on breathing and respiratory diseases" was published in 2009. Journal: Lung India.

Sleep study should be evaluated in patients with primarily non-respiratory conditions, similar to patients who are prone to cerebrovascular or cardiovascular diseases and identify any underlying respiratory insufficiency increasing risk of the disease. It may then be a helpful tool in management and treatment of patients suffering from the above-mentioned diseases.
